The article "Research on Nanoeffect of Penetration and Consolidation under Nonlinear Characteristics of Saturated Soft Clay" was retracted in 2023. Reasons: signs of a paper mill; compromised peer review; unreliable results or conclusions.

# Research on Nanoeffect of Penetration and Consolidation under Nonlinear Characteristics of Saturated Soft Clay

**DOI:** 10.1155/2022/7463817

**Published:** 2022-06-02

**Authors:** Yu Zhao, Ning Wang, Deying Zhang

**Affiliations:** College of Civil Engineering, Shijiazhuang Tiedao University, Shijiazhuang, Hebei 050043, China

## Abstract

In order to systematically study the nanopermeability properties of saturated soft clay under different consolidation pressures and different osmotic pressures, this paper analyzes various loading and unloading conditions that affect the permeability of soil based on the material description equation with displacement as the control variable of large deformation consolidation theory. By summarizing the empirical relationship between permeability coefficient and consolidation pressure and permeability coefficient and void ratio, the infiltration law and seepage failure characteristics of soft clay are revealed. For the soil studied in this paper, a = 0.65, *b* = 0.001, and *q* = 3.55 are acceptable. The effect of the initial permeability coefficient on large deformation consolidation is studied, and the necessity and plausibility of considering the nonlinearity of the compression and permeability coefficient when calculating the soft-land base large deformation consolidation is also studied.

## 1. Introduction

Since the advent of Darcy's law, the study of soil permeability has experienced a long time. Studies have shown that Darcy's law for describing the saturated sand under the laminar state seepage is very successful, but due to the applicability of clayey soil in different understanding, many scholars through experiments discovered the clayey soil seepage law of Darcy off [1]. For example, in terms of research ideas, the comprehensive effects of gravity water, capillary water, and weakly binding water under the action of different hydraulic gradients have been considered, the structure of cohesive soil has been considered, and the permeability coefficient of rock and soil mass has been regarded as a random variable to analyze the seepage condition of the soil layer, etc. [2, 3]. Some studies have been improved continuously from the aspect of test instruments. For example, the improved triaxial apparatus, the GDS consolidation test system, the HS2K-0L permeability coefficient rapid test system, etc. In addition, there are some differences in academic circles about whether there is an initial hydraulic slope for clay soil and how to consider it in practice [4, 5]. Although the reason for the existence of an initial hydraulic slope can be explained mechanically, many early tests on undisturbed soil have proved that this minimum hydraulic slope is not obvious. Although many experiments have confirmed the existence of initial hydraulic slope for seepage in clay soils, there is no consensus on how to apply this result to consolidation theory and current regulations.

In the 1950s and 1960s, scholars began to use model theory to describe the rheological properties of soil; that is, several linear spring elements combined with linear or nonlinear clay pot elements were used to describe the constitutive relationship of soil. Chen Zongji was the first scholar in China who introduced rheology theory into the field of consolidation settlement. He proposed a consolidation theory based on the assumption that the soil skeleton was viscoelastic [6]. M. Kotilek summarized 12 kinds of NON-Darcy V-I relations and believed that the experimental method and errors in the experimental process were the main reasons for the deviation of the seepage law from Darcy's law. Zhang Zhong explained the deviation phenomenon from the perspective of bound water and believed that the non-Darcy seepage in clay was due to the non-Newtonian behavior of pore water [7]. L. Erge believed that whether Darcy's law applies to clay should be further discussed [8]. Wang Xiuyan et al. believed that the seepage law of saturated clay should be discussed through other paths. He believed that secondary consolidation was caused by the following reasons: (1) viscous shear flow due to deviant stress; (2) viscous volume flow due to spherical stress; the hysteresis of volumetric deformation is not only caused by the viscoelastic property of soil skeleton itself but also by the hysteresis of pore water extrusion; (3) when the above two flows occur, hardening also occurs. However, since Chen Zongji considered extending the theory to three-dimensional problems at the beginning of establishing the theory, it was difficult to determine the parameters and it was too complicated to apply it to one-dimensional problems. As for the pore pressure of soft clay under cyclic loading, Seed and Chen believed that rectangular wave load had a greater effect than triangular wave load [9, 10]. Shibata also believes that rectangular wave load has greater influence than sinusoidal wave load. Se and Chan studied the influence of different loading durations and intervals on the deformation characteristics of silty sand and silty clay [11]. They believe that when the loading interval is more than 2 minutes, the larger the loading duration is, the larger the deformation will be. For silty clay, the deformation is not always proportional to each loading duration but may increase or decrease with the loading duration. Deformation may also increase or decrease, depending on the loading interval. Since the osmotic consolidation process of saturated clay is a process of continuous drainage of pore water, the seepage law will affect the process of osmotic consolidation [12, 13]. Literature has discussed the influence of initial hydraulic gradient on one-dimensional consolidation of saturated clay, and it is believed that the average consolidation rate of clay is slower than Terzaghi's theoretical value of one-dimensional consolidation [14]. The Hansbo seepage model is introduced into the consolidation analysis of saturated clay in the literature, and studies show that such nonlinear seepage slows the dissipation rate of pore water pressure in saturated clay [15, 16]. Therefore, it is very important to discuss the form of seepage and the variation of its parameters in saturated clay for further exploring the mechanism of seepage consolidation in saturated clay. Because the traditional permeability test cannot get the change law of permeability coefficient in the consolidation process and cannot study the non-Darcy seepage form, its parameters, and the consolidation pressure with the change of pore ratio in the consolidation process, the author improved the traditional consolidation permeability test device and designed a new consolidation permeability test. The permeability characteristics of saturated clay under different consolidation pressures were studied [17].

In this paper, according to the existing research results on saturated cohesive soil permeability law, combined with the engineering properties of soil, the permeability characteristics of saturated cohesive soil under different consolidation pressures and different seepage pressures are studied through laboratory permeability tests. Based on the large deformation consolidation theory and the material description equation with displacement as the control variable, the influence of clay permeability on large deformation consolidation is analyzed.

## 2. Research Methods

### 2.1. Experimental Study on Permeability Characteristics

#### 2.1.1. Test Scheme

The test was carried out on an STOY-3 osmotic pressure tester. During the test, consolidation pressure was first applied according to the requirements, and the variable head osmotic pressure test was carried out after the corresponding consolidation of soil samples was completed. The test object is gray-black undisturbed soft clay with a depth of 4∼6m and a small amount of sand. The basic physical and mechanical properties of the soil samples are shown in Table 1.

Table 2 shows the test scheme of permeability characteristics (test head ‰ > 2.0 m) in which the osmotic pressure P′ is applied by air compressor, and the conversion relationship between P′ and head h0 is h0 = *γ*_w_

### 2.2. Influence of Permeability Characteristics on One-Dimensional Large Deformation Consolidation

#### 2.2.1. Approximate Analytical Solution of Large Deformation Consolidation Equation

One-dimensional large deformation consolidation equation with displacement as control variable in solid phase coordinates can be expressed as follows:

(1) $$\begin{array}{c} \frac{\partial u}{\partial t}=c^{2}\frac{\partial^{2}u}{\partial z^{2}}-A\left(0<z<l_{0},k\;t>0\right),\\ u|{}_{t=0}=0,\\ u|{}_{z=0}=0,\\ \frac{\partial u}{\partial t}|{}_{z=l_{0}}=a, \end{array}$$

where z is the vertical solid coordinate (positive upward); t is the initial thickness of soil; *c*^2^=_*C*_*v*0__*B*=_*C*_*v*0__(1+*∂u*/*∂z*)^−3^; *C*_*v*0_=*k*_0_*E*_*s*_/*γ*_*w*_; Es is the compressibility parameter of soil, which can be expressed as the comparison value of stable void ratio and initial void ratio of soil: *A*=*k*(*γ*_*s*_ − *γ*_*w*_)/*γ*_*w*_(1+*e*_0_); is the surface displacement gradient under the action of external load g; and *α*=(2*q*/*E*_*s*_+1)^2^ − 1. When b is a constant, the analytical solution of formula can be obtained by the method of separating variables as follows:

(2) $$\begin{array}{c} u\left(z,t\right)=\frac{A}{2c^{2}}z^{2}+\left(\alpha +\frac{Al_{0}}{c^{2}}\right)z+2\left(\frac{Al_{0}}{c^{2}}-\alpha \right)l_{0}\\ \sum_{n=1}^{\infty }\frac{\sin\;M}{M^{2}}\exp\left[-{\left(\frac{M_{c}}{l_{0}}\right)}^{2}t\right]\sin\left(\frac{M_{z}}{l_{0}}\right)\\ \left(M=\left(2n-1\right)\frac{\pi }{2},\;n=1,2,3,...\right). \end{array}$$

If *A* = 0 is assumed, the formula is simplified as a consolidation solution ignoring the self-weight of soil. When *B* = 1 is further assumed, the equation degenerates into consolidation solution under linear elastic small strain.

## 3. Research Results

### 3.1. Influence of Consolidation Pressure and Osmotic Pressure on Permeability Characteristics

The loading proportional coefficient is L = Pc/Pi (where Pi is the first consolidation pressure). Considering the preconsolidation pressure, it is determined for the test soil sample that which is ≈80kPal.

Figure 1 shows the relationship curve between loading proportional coefficient and permeability coefficient obtained from experiments. It can be seen from Figure 1 that the permeability coefficient k decreases with the increase of loading ratio l and tends to be stable gradually. It shows that when the consolidation pressure reaches a certain value, the pore channels of soil will be compressed to a certain critical value. Further compression is mainly due to the compression of soil aggregates and the reorientation of particles inside the aggregates, and the influence on permeability is negligible. In addition, with the increase of consolidation pressure, the pore channels gradually become smaller, and the viscous resistance of bound water in the soil will continue to increase, thus forming a “relatively stable” state in which the k-L curve decreases slightly but is basically flat in the second half.

Figure 2 shows the relationship diagram of seepage velocity-consolidation pressure-seepage pressure (v-p-p') under higher water head (*h*0 > 2m), which further reflects the seepage characteristics of soil under consolidation pressure. The seepage velocity decreases with the increase of consolidation pressure, showing a nonlinear inverse relationship. When the consolidation pressure reaches a certain value, the seepage tends to be stable due to the compaction of soil, and the seepage velocity is a smaller value. V-p' is linear, slope can reflect the seepage state of soil under corresponding consolidation pressure, and seepage pressure (p') has an obvious effect on the linear increase of seepage velocity.

The test results in Figure 3 show that the permeability coefficient is mainly related to the current stress state and is not affected by the consolidation path.

Because the consolidation pressure changes the pore channel and the structure of soil, the smaller pore channel makes the resistance effect of bound water more obvious. When the pore diameter is compressed to have little difference with the thickness of bound water film, the viscous resistance of the bound water will seriously hinder the flow of water in soil and greatly reduce the permeability characteristics of soft clay. Therefore, the permeability characteristics of saturated soft clay are mainly affected by consolidation and compaction, and the permeability law obeys Darcy's Law of Permeability under higher water head [18, 19]. When the consolidation state of soil reaches a stable state, the seepage velocity of pore water tends to a “stable state”. According to the test results, the consolidation pressure corresponding to this stable value is 4∼5 times the preconsolidation pressure.

### 3.2. Influence of Permeability Characteristics on Large Deformation Consolidation

E-p and k-p empirical formulas (*e*(P) = 1/(a + bp) and *k*€ = k0exp (Q(e-e0))) obtained from the previous permeation test are substituted into a and c in the above formula, and the test parameters are a = 0.65 and *b* = 0.00 l. In order to consider the different permeability coefficients of different soil depths, *p*=*q*+∑_*i*=1_^*n*^*γ*_*i*_(*h*_*i*_ − *z*_*i*_), where q in the e-p relationship is the external load of the surface and h_i_ and Yi are the thickness and gravity of each layered soil of foundation, respectively. Choose the case of large area load acting on a homogeneous foundation as shown in Figure 4 and solve it by Matlab programming. The deformation of the soil layer under various conditions can be obtained.  Figure 5 shows the calculation results with different initial permeability coefficients k0.

In Figure 5, *z* = 10 m indicates the top of the compression layer, and the maximum consolidation time is 2a. The results show that k0 has an influence on surface settlement, foundation consolidation displacement, and foundation consolidation depth. Increasing soil permeability can accelerate soil consolidation and deepen consolidation depth, but more calculation comparisons show that this influence is related to the initial void ratio e0 and overlying load. When e0 is constant there is a critical value for the influence of k0. When the overlying pressure Q increases, the significance of this effect will increase.  Figure 6 shows the calculation results of large deformation consolidation by using the theory of large deformation consolidation but without considering the nonlinearity of *k* and *e*, i.e. *k* = *k*0 and *e* = *e*0 in the formula. Compared with Figure 5, the consolidation displacement and the consolidation depth increase at the same time t. And the calculation shows that the difference will further increase in the later stage of consolidation.

Because the consolidation delay of deep soft soil will affect the transmission and change of effective stress in the consolidation process, and because it has the mechanical characteristics of material nonlinearity, if the change of permeability coefficient with compressibility is not considered when considering the geometric nonlinearity of soil deformation, the calculation results cannot fully reflect the essential difference between large deformation consolidation theory and small deformation consolidation theory. This is especially true when the load level is large. Only when the thickness of soil layer is thin, the permeability of the soil is good, or the load level is low is the calculation result without considering the change of permeability coefficient is considered reasonable, but in this case, the large deformation consolidation theory can be omitted [20]. So, the nonlinear variation of permeability coefficient with soil compressibility must be considered when a large deformation consolidation calculation is adopted. By integrating small deformation calculation methods such as the final settlement estimation method, layered summation method, and Karl Terzaghi consolidation equation with large deformation consolidation equation, it is found that when the soil surface load is not large, the difference of final settlement calculated by various methods is small, and this difference increases with the increase of soil surface load, which gradually shows that the result obtained by the large deformation algorithm is smaller than the result calculated by Karl Terzaghi but similar to the layered summation method. This conclusion is consistent with Xie Xinyu's research results. In addition, The calculation results also show that the consolidation settlement obtained by the Karl Terzaghi algorithm has an obvious lag.

Because the deformation of soft clay under consolidation pressure is mostly reflected as unrecoverable deformation, the permeability coefficient will not recover with the unloading rebound of soil. Saturated cohesive soil does have the phenomenon that the initial hydraulic gradient and the seepage law deviate from Darcy's law when the hydraulic gradient is low, so the influence of the initial gradient should be considered in the test method. According to the hydraulic gradient, the infiltration law can be described by adopting the method of obeying Darcy's law in sections or simply adopting *v*=*k*(i-i0). In addition, the seepage failure mode of soft clay is related to consolidation pressure.

## 4. Conclusions

The permeability coefficient k decreases with the increase of overlying consolidation pressure and gradually tends to a stable value with the increase of consolidation pressure, satisfying the relationship of *k* = c/(aL + b). Infiltration velocity decreases with the increase of consolidation pressure, showing a nonlinear inverse relationship. Seepage velocity and osmotic pressure show a linear relationship. The permeability coefficient is mainly related to the current stress state and is not affected by the consolidation path. The relationship between permeability coefficient and porosity ratio and the relationship between porosity ratio and consolidation pressure can be expressed as *k*(*e*)=*k*_0_exp⌊*Q*(*e* − *e*_0_)⌋ and *e*(p) = 1/(a + bp) mathematical models, respectively, and the parameters in the models can be determined by an osmotic pressure test. For the soil studied in this paper, *A* = 0.65, *B* = 0.001, and *Q* = 3.55 can be adopted.

In the calculation of large deformation consolidation, the consolidation displacement and the depth of soil layer at time t are related to the initial permeability coefficient k0, but under certain conditions of e0, the influence of k0 has a critical value, and when the overlying pressure q increases, the significance of the influence will increase. For deep soft soil foundation, if the nonlinearity of K and E is not considered in the calculation of large deformation consolidation, at the same time, both the consolidation displacement and the consolidation depth will increase, but the calculation results cannot fully reflect the essential difference between the large deformation consolidation theory and the small deformation consolidation theory, especially when the load level is high.

## Figures and Tables

**Figure 1:** L Relationship curve between loading proportional coefficient and permeability coefficient.

**Figure 2:** V-p-p' relationship under different loading conditions.

**Figure 3:** Relationship between permeability coefficient and consolidation pressure under different consolidation paths.

**Figure 4:** Schematic diagram of soft soil foundation.

**Figure 5:** The influence of *k*0 on large deformation consolidation when *k* = *k* (e) (*e* = 1.54). (a) *k*_0_ = 3.6 ∗ 10^−7^ cm/s. (b) *k*_0_ = 3.6 ∗ 10^−6^ cm/s.

**Figure 6:** Calculation results of large deformation consolidation (*k* = *k*_0_, *e* = *e*_0_). (a) *k*_0_ = 3.6 ∗ 10^−7^ cm/s. (b) *k*_0_ = 3.6 ∗ 10^−6^ cm/s.

**Table 1:** Physical and mechanical properties of soil samples.

*W* (%)	*ρ* (g*∗*cm^−3^)	ds	*e*	Sr (%)	wL (%)	wp (%)	Ip	IL	al-2 (MPa^−1^)	Consolidation quick shear *φ*/(*o*)*c*/kPa		*K*_0_ (10^−8^ cm *∗* s^−1^)
54.5	1.68	2.72	1.54	96.3	52.3	19.5	32.8	1.1	1.29	17.5	8.9	7.25

**Table 2:** Test scheme of permeability characteristics.

Experimental scheme	Loading (unloading) stress path
Different consolidation pressures p	50-100-200-300-400 kPa
Different osmotic pressures *P*′	The consolidation path is 50-100-200-300-400 kpa, and the osmotic pressure p′ = 20,30,50,75, 100 kPa is applied under each stage of consolidation.
Add lotus	50-100-200-300-400 kPa
	50-100-200–400 kPa
Different consolidation paths	50–400 kPa
	50-200-400–800 kPa
	50-400-800 kPa
unload	100-75-50-25-0 kPa
lotus	200-150-120-100-50 kPa
Different initial consolidation pressures	300-200-150-100-50 kPa
p_max_ and different unloading paths	400-200-100-50-0 kPa
	800-400-200-100-50-0 kPa
	50-100-200-300-400-200-50 kPa

## Data Availability

The data used to support the findings of this study are available from the corresponding author upon request.

## References

[1] Lu Y., Liu F., Bian Y., Zhong Y., Chen B., Huang J. (2020). Dynamic chikaracteristics of saturated soft clay under constant confining pressure cyclic loading. *IOP Conference Series: Earth and Environmental Science*.

[2] Yang D., Li F., Xia Y., Shi M., Hao Y. (2021). Analysis of elastic viscoplastic consolidation of sand drain foundations with exponential seepages. *E3S Web of Conferences*.

[3] Li C. X., Dong X. Q., Jin D. D., Xie K. H. (2017). Nonlinear large-strain consolidation analysis of soft clay considering threshold hydraulic gradient. *Yantu Lixue/Rock and Soil Mechanics*.

[4] Kosterin A. V., Skvortsov é. V. (2018). Seepage consolidation under plane deformation of elastic half-space. *Fluid Dynamics*.

[5] Xu C., Wang X., Lu X., Da I F., Jiao S. (2018). Experimental study of residual strength and the index of shear strength characteristics of clay soil. *Engineering Geology*.

[6] Dai G.-l., Zhu W.-B., Gong W. M., Zhai Q., Zhao X.-l. (2020). Characteristic test study on bearing capacity of suction caisson foundation under vertical load. *China Ocean Engineering*.

[7] Chittoori B. C. S., Moghal A. A. B., Pedarla A., Al-Mahbashi A. M. (2017). Effect of unit weight on porosity and consolidation characteristics of expansive clays. *Journal of Testing and Evaluation*.

[8] Saisubramanian R., Murugaiyan V., Sundararajan T. (2019). Studies on characteristics, applications and strength improvement of marine clay: a review. *Journal of Geoscience and Environment Protection*.

[9] Wang Y., Li X., Lan R., Ning W., Chen H. (2017). Development and prospect of study on soil nonlinear dynamic characteristics under strong-motion. *Earthquake Research in China*.

[10] Dai J., Su Z., Zhao M., Xiang Y. (2017). True triaxial tests on stress-strain characteristics of soft clay considering the structural effects. *Yanshilixue Yu Gongcheng Xuebao/Chinese Journal of Rock Mechanics and Engineering*.

[11] Yang A. W., Kong L. W., Guo F. (2017). Accumulative plastic strain characteristics and growth model of tianjin binhai soft clay under cyclic loading. *Yantu Lixue/Rock and Soil Mechanics*.

[12] Zhu W. L., Chang H., Zhao S. Y. (2021). Model test on bearing capacity characteristics of energy piles in saturated clay. *IOP Conference Series: Earth and Environmental Science*.

[13] Liu G., Xie Q., Fan G., Qian F., Qi C. (2017). Model test on bearing capacity characteristics of heat exchanger piles in saturated clays. *Yanshilixue Yu Gongcheng Xuebao/Chinese Journal of Rock Mechanics and Engineering*.

[14] Wang Y., Cai Z., Cai Y., Guan Y., University N., Department G. E. (2017). Comparative studies of creep characteristics of saturated soils at drained k_0 consolidation. *Journal of Basic Science and Engineering*.

[15] Shi G., Liu Z. Y., Li Y. H. (2018). One-dimensional rheological consolidation of soft clay under cyclic loadings considering non-Darcy flow. *Yantu Lixue/Rock and Soil Mechanics*.

[16] Zou S. F., Li J. Z., Wang Z. J., Lan L., Xie X. Y. (2017). Seepage test and empirical models for soils based on gds apparatus. *Zhejiang Daxue Xuebao (Gongxue Ban)/Journal of Zhejiang University*.

[17] Li C. X., Xiao J., Yang Y., Wu W. (2018). One-dimensional large-strain nonlinear consolidation of overconsolidated clays with a threshold hydraulic gradient. *Advances in Civil Engineering*.

[18] Rusdiansyah (2021). The effect of temperature on the engineering properties consolidation behaviors of soft soil. *Istrazivanja i Projektovanja za Privredu*.

[19] Li Y., Zhang K., Hu H., Nie S. (2017). The characteristics of microstructure change of sand grain mucky soil under different consolidation pressures. *Modelling, Measurement & Control, C*.

[20] Huang Y., Li T., Fu X. (2021). Consolidation of unsaturated drainage well foundation with smear effect under time-dependent loading. *KSCE Journal of Civil Engineering*.

